RETRACTED

# Modulatory Role of PYY in Transport and Metabolism of Cholesterol in Intestinal Epithelial Cells

**DOI:** 10.1371/journal.pone.0040992

**Published:** 2012-07-23

**Authors:** Emilie Grenier, Carole Garofalo, Edgard Delvin, Emile Levy

**Affiliations:** 1 Research Centre, Centre Hospitalier Universitaire (CHU) Ste-Justine, Montreal, Quebec, Canada; 2 Department of Nutrition, Université de Montréal, Montreal, Quebec, Canada; 3 Department of Biochemistry, Université de Montréal, Montreal, Quebec, Canada; National Institute of Agronomic Research, France

## Abstract

**Background:**

Gastrointestinal peptides are involved in modulating appetite. Other biological functions attributed to them include the regulation of lipid homeostasis. However, data concerning PYY remain fragmentary. The objectives of the study were: (i) To determine the effect of PYY on intestinal transport and synthesis of cholesterol, the biogenesis of apolipoproteins (apos) and assembly of lipoproteins and (ii) To analyze whether the effects of PYY are similar according to whether cells are exposed to PYY on apical or basolateral surface.

**Methodology/Principal Findings:**

Caco-2/15 cells were incubated with PYY (1–36) administered either to the apical or basolateral medium, at concentrations of 50 or 200 nM for 24 hours. *De novo* synthesis of cholesterol, cholesterol uptake, and assembly of lipoproteins were evaluated through the incorporation of [^14^C]-acetate, [^14^C]-cholesterol, and [^14^C]-oleate, respectively. Biogenesis of apos (A-I, A-IV, E, B-48 and B-100) was examined by the incorporation of [^35^S]-methionine. The influence of PYY on protein and mRNA levels of many key mediators of lipid metabolism was analyzed by Western blot and PCR, respectively. Our results show that PYY influenced cholesterol metabolism in Caco-2/15 cells depending on the site of PYY delivery. Apical addition of PYY significantly lowered the incorporation of [^14^C]-cholesterol likely via the reduction of NPC1L1, stimulated intracellular cholesterol synthesis probably through an increase in SREBP-2 expression, whereas it concomitantly increased apo A-I synthesis and decreased LDL secretion. In contrast, basolateral PYY reduced the production of chylomicrons (CM) as well as the biogenesis of apos B-48 and B-100, while lowering the expression of the transcription factors RXRα and PPAR(α,β).

**Conclusions/Significance:**

PYY is capable of influencing cholesterol homeostasis in intestinal Caco-2/15 cells depending on the site delivery. Apical PYY was able to decrease cholesterol uptake via NPC1L1 downregulation, whereas basolateral PYY diminished CM output through the biogenesis decline of apos B-48 and B-100.

RETRACTED

## Introduction

Peptide YY (PYY), a 36 amino acid straight chain polypeptide, is produced by epithelial entero-endocrine L cells throughout the gut, but its concentrations increase distally, reaching higher levels in the colon and rectum [1], [2]. The predominant form of PYY is released into the circulation as PYY(3–36), with the Nterminal truncated by the enzymatic action of dipeptidyl peptidase (DPP-IV) [3], [4]. Peptide YY(3–36) is secreted in proportion to the amount of calories in the meal, with serum concentrations increasing within 15 min of a meal, peaking at about 60 min and sustaining for up to 6 h [5]. The secretion is mediated by neural reflex and by direct contact of nutrients; however, fat intake promotes higher secretion of PYY(3–36) than carbohydrates and proteins [6].

Although PYY is localized in mucosa, it may act as an endocrine modulator of distant target tissues, particularly within the gastrointestinal tract. In fact, PYY exhibits various actions on this tissue, including the delay of both gastric emptying and mouth to caecum transit time [7], the inhibition of jejunal pressure wave activity [8], the reduction of pentagastrin-stimulated acid secretion [6], the cephalic phase related to negative pancreatic exocrine secretion in man [9]–[11], and actin arrangement and expression of cytoskeletal proteins in intestinal epithelial cells, which interact with organizing intracellular structure, such as cellular-extracellular matrix [12]. This regulation by PYY enhances the efficiency of nutrient digestion and absorption, and ensures efficient utilization of ingested food. Furthermore, PYY can initiate an “ileal brake” when the rate of triglyceride (TG) hydrolysis exceeds the rate of fatty acid (FA) absorption excess [10], [13], [14]. In addition, PYY interacts with FAs to induce differentiation in mucosal cells [15], [16].

As reported above, PYY modulates important gastrointestinal functions with important effects on food intake and energy expenditure, which influences the delivery of nutrients and gut hormones to the circulation. There is also evidence that PYY is closely involved in insulin secretion and glucose homeostasis [17]. Furthermore, peripheral administration of PYY has been shown to increase blood pressure in healthy humans [18], which suggests that this gut hormone may also influence cardiovascular diseases in addition to modulating appetite and metabolism. Accordingly, recent studies have reported an inverse correlation between fasting PYY and total cholesterol [19], as well as low- and high-density lipoprotein cholesterol levels [20], which indicates that the PYY gut hormone may be involved in the modulation of cholesterol metabolism. Intriguingly, the role of PYY in intestinal cholesterol transport has not been investigated. Therefore, the major aim of this study is to determine whether PYY is able to modulate intestinal cholesterol synthesis, apolipoprotein (apo) biogenesis and lipoprotein assembly and secretion. These issues were tackled using the Caco-2/15 cell line that spontaneously differentiates into polarized mature enterocytes under standard culture conditions, and lends itself to the in *vitro* study of human gut in view of its efficient intestinal transport processes [21].

RETRACTED

With Caco-2/15 cells granting access to both apical and basolateral sides of the bipolar intestinal epithelium when cultured on Transwell filters, we were also able to underline the importance of the regulatory site of intestinal cholesterol transport by PYY since this gastrointestinal factor was found to be secreted in the two compartments [22]–[25].

## Materials and Methods

### Cell Culture

The human epithelial colorectal adenocarcinoma Caco-2/15 cell line, a stable clone of the parent Caco-2 cells (American Type Culture Collection, Rockville, MD), was obtained from Dr. JF Beaulieu (Department of Cellular Biology, Faculty of Medicine, Université de Sherbrooke, Sherbrooke, Quebec, Canada) [26]–[28]. Caco-2/15 cells were grown at 37°C with 5% CO_2_ in MEM (GIBCO-BRL, Grand Island, NY) containing 1% penicillin-streptomycin and 1% MEM nonessential amino acids (GIBCO BRL) and supplemented with 10% decomplemented fetal bovine serum (FBS) (Flow, McLean, VA) as described previously [29]. Caco-2/15 cells (passages 30–40) were maintained in T-75-cm^2^ flasks (Corning Glass Works, Corning, NY). Cultures were split (1∶6) when they reached 70–90% confluence, by use of 0.05% trypsin-0.5 mM EDTA (GIBCO-BRL). For individual experiments, cells were plated at a density of 1×10^6^ cells/well on 24.5-mm polycarbonate Transwell filter inserts with 0.4-µm pores (Costar, Cambridge, MA), in MEM (as described above) supplemented with 5% FBS. The inserts were placed into six-well culture plates, permitting separate access to the apical and basolateral compartments of the monolayers. Cells were cultured for 14 days at which the Caco-2/15 cells are highly differentiated into polarized mature enterocytes and appropriate for lipid metabolism [29], [30]. The medium was refreshed every second day.

### PYY (1–36)

Human PYY (1–36) (Sigma) was added to cells in apical or basolateral compartments at different concentrations (50 nM or 200 nM) for 24 h.

### Isolation of Apical or Basolateral Membranes from Differentiated Caco-2/15

14 days after reaching 100% confluence until fully differentiated, the brush border fractions were prepared by a modification of the method of Schmitz et al. [31]. Briefly, the culture medium was removed, and the cells were rinsed twice with Phosphate Buffer Saline (PBS, GIBCO-BRL). The cells were homogenized in 50 mM mannitol-HCL solution, pH 7.5, supplemented with 0.15 mg/ml leupeptin, 100 U/ml trasylol, 1×10^−13^ mg/ml pepstatin, and 1 mM PMSF. After the addition of CaCl_2_ to a final concentration of 10 mM, the homogenate was centrifuged for 15 min at 5000×*g* and 4°C to provide a pellet containing basolateral membrane. The supernatant was subsequently centrifuged first for 20 min at 30000×*g* and 4°C and then for 30 min at 30000×*g* and 4°C. The final pellet containing the apical membranes was frozen.

RETRACTED

### Cholesterol Absorption by Caco-2/15 Cells

Cholesterol uptake by the cells was assessed following its solubilisation in albumin as described previously [32], [33]. The differentiated cells were incubated at 37°C for 24 h in MEM containing 50 nM or 200 nM of PYY, in apical or basolateral compartments, as well as cholesterol solution added to the apical medium. At the end of the treatment, cells were washed twice with cold PBS (sufficient to complete removal of labelled cholesterol bound on cell membranes as established in our laboratory by various methods such as cyclodextrin), scrapped in 1 ml lysis buffer (5 mM Tris, 15 mM NaCl, EDTA 5 mM, 0.1% SDS, 1% Triton×100, 0.5% sodium deoxycholate) and homogenized by sonication followed by a 5 min at 13800×g centrifugation to remove cell debris. An aliquot of 0.1 ml was placed in a scintillation vial with Ready Safe counting fluid (Beckman, Fullerton, CA). Radioactivity was measured by scintillation counting (LS 5000 TD, Beckman). Cell protein was quantified by the Bradford method (BioRad).

### Lipid Carrier

Blood (20 mL) was collected by venipuncture 2–3 h after the ingestion of a high fat meal (50 g/1,73 m^2^) from two human healthy volunteers. This procedure was approved by the Institutional Ethic Committee. After a 1000×g centrifugation to pellet red blood cells, postprandial plasma was supplemented with 1 mM of aprotinin and 0.1% of sodium azide and was mixed with basolateral media to serve as a carrier for the isolation of labeled chylomicron (CM) as described previously [29].

### *De novo* Lipogenesis

Caco-2/15 cells were serum-starved after 14 days of differentiation on Transwell filter inserts. After 18 h-incubation in serum-free medium, cells were cultured in the presence of 5 µCi of sodium-[^14^C]-acetate (specific activity of 50–62 mCi/mmol; GE Healthcare, Piscataway, NJ) for 24 h. Cells and media were collected, supplemented with a mixture of anti-proteases and lipids were extracted overnight in chloroform-methanol (2∶1, vol:vol). Lipids recovered were separated on TLC plates, and bands corresponding to free cholesterol and cholesteryl ester were scraped off the plates, mixed with scintillation fluid and counted for the amount of radioactivity incorporated as described previously [34].

RETRACTED

### Isolation of Lipoproteins

Radiolabeled [^14^C]-oleic acid (sp act, 53 mCi/mmol, Amersham, Oakville, ON, Canada) was added to unlabeled oleic acid and then solubilised in FA-free bovine serum albumin (BSA) [BSA/oleic acid, 1∶5 (mol:mol)]. The final oleic acid concentration was 0,7 mM (0,45 µCi)/well. Cells were first washed with PBS, and the [^14^C]-oleic acid-containing medium was added to the apical compartment. PYY (1–36) was added to the apical and basolateral chamber in serum-free MEM. At the end of a 24 h incubation period, cells were washed and then scraped with a rubber policeman in a PBS solution containing antiproteases (phenylmethylsulfonyl fluoride, pepstatin, EDTA, aminocaproic acid, sodium azide and trasylol, all at a final concentration of 1 mM). The medium was first mixed with a plasma lipid carrier (4∶1, vol/vol) to efficiently isolate de novo lipoproteins synthesized.

The lipoproteins were then isolated from basolateral media by serial ultracentrifugation using a TL-100 ultracentrifuge (Beckman-Coulter, Fullerton, CA) according to the method described previously [35]. Briefly, CM were first isolated after an ultracentrifugation (20000 rpm for 20 min). Very-low density lipoprotein (VLDL; 1.006 g/mL) and low density lipoprotein (LDL; 1.063 g/mL) were subsequently separated by centrifugation at 100000 rpm for 2.5 h with a tabletop ultracentrifuge 100.4 rotor at 4°C. The High density lipoprotein (HDL) fraction was obtained by adjusting the LDL infranatant to density at 1.21 g/mL and centrifuging for 6 h at 100000 rpm. Each lipoprotein fraction was exhaustively dialyzed against 0.15 M NaCl and 0,001 M EDTA, pH 7.0 at 4°C for 24 h.

### De novo Apolipoproteins Synthesis and Secretion

The effect of PYY (1–36) on newly synthesized apos (A-I, A-IV, B-48, B-100 and E) was assessed as described previously [29]. To induce apo synthesis, cells were incubated apically with unlabeled oleic acid bound to albumin in serum-free medium, 18 h before [^35^S]-methionine incubation. Thereafter, cells as well as the outer chambers were rinsed twice with PBS. The apical compartment was replaced with 1.5 ml of methionine-free medium containing the unlabeled substrate (oleic acid) and 100 µCi/ml [^35^S]-methionine (50 mCi/mmol, Amersham Life Sciences). During this time, PYY (1–36) (Sigma) was added to the apical or basolateral chamber. Following basolateral medium removal, cells were scraped off the inserts in the cell lysis buffer. The cell lysates and media were supplemented with an antiprotease cocktail and analysed for apo synthesis and secretion, respectively, using antibodies with high specificity, which was tested by assessing cross reactivity, the recognition of a specific apo among a cocktail of various proteins, and the use of control conditions (omission of antibodies or exclusive treatment with pre-immune rabbit sera).

RETRACTED

### Immunoprecipitation of Apolipoproteins

Immunoprecipitation of apos in cell lysates and basolateral media was performed in the presence of excess polyclonal antibodies to human apos (A-I, A-IV, E, with a dilution of 1/1000; Santa Cruz, CA) and apo B (with a dilution of 1/1000; Boehringer, Mannheim) overnight at 4°C. Samples were then washed with lysis buffer. They were subsequently centrifuged and resuspended in sample buffer (1.2% SDS, 12% glycerol, 60 mM Tris, pH 7.3, 1.2% β-mercaptoethanol, and 0.003% bromophenol blue) and analyzed by a linear 4–15% polyacrylamide gradient preceded by a 3% stacking gel. Radioactive molecular weight standards (Amersham Life Sciences) were run in the same conditions. Gels were sectioned into 2-mm slices and counted after an overnight incubation with 1 ml of Beckman tissue solubilizer (0.5 N quaternary ammonium hydroxide in toluene) and 10 ml of liquid scintillation fluid (Ready Organic, Beckman). Results for each apo studied were expressed as percent disintegrations per minute per milligram protein to assess the specific effect of PYY (1–36) on apo synthesis.

### Western Blot

To assess the presence of Niemann-Pick C1 like 1 (NPC1L1), Scavenger receptor-class B type I (SR-BI), CD36, ATP binding cassette subfamily (ABCG5, ABCG8), LDL-receptor (LDL-R), HMG-CoA reductase (HMG-CoA-R), Acyl-Coenzyme A:cholesterol acyltransferase (ACAT)-2, and microsomal triglyceride transfer protein (MTP), Caco-2/15 cells were homogenized and prepared for Western blotting. The Bradford assay (Bio-Rad) was used to determine protein concentration. Proteins were denatured in sample buffer containing SDS and β-mercaptoethanol, separated on a 7.5% SDS-PAGE gel, in the presence of a cocktail of a high-range rainbow molecular weight markers (myosin, 220, 000 Da; phosphorylase b, 97,000 Da; BSA, 66,000 Da; ovalbumin, 45,000 Da; carbonic anhydrase 30,000 Da; trypsin inhibitor, 20,100 Da; Lysozyme, 14,300 Da from GE Healthcare) and blotted onto nitrocellulose membranes. Purified apos also served as markers for apo mobility. Nonspecific binding sites of the membranes were blocked with 5% defatted milk proteins. Reactions took place by the addition of primary antibodies directed against targeted proteins: NPC1L1 (1/3000; Novus), SR-BI (1/50000; Novus), CD-36 (1/5000; Santa Cruz), ABCG5 (1/1000; Santa Cruz), ABCG8 (1/500; Novus), LDL-R (1/20000; Fitzgerald), HMG CoA-R (1/10000; Upstate), phosphorylated (P)-HMG CoA-R (1/10000; Millipore), ACAT-2 (1/5000; Cayman), and MTP (1/3000; Provided by Dr. David Gordon, Bristol-Myers-Squibb). Reaction was revealed with species-specific horseradish peroxidise-conjugated secondary antibody (1/20000; Roche Diagnostic, Mannheim) for 1 h at room temperature. β-actin (with Ab dilution of 1/5000) was used as an internal control to confirm equal loading protein on SDS-PAGE. Blots were developed with the chemiluminescent substrate Luminol (Roche) and proteins were quantified by use of a Hewlett-Packard scanner equipped with a transparency adaptor and UN-SCAN-IT (Silk Scientific) software.

RETRACTED

### RT-PCR

PCR experiments for the various genes [(liver X receptors (LXRs); retinoid X receptors (RXRs); peroxisome proliferator-activated receptors (PPARs) and sterol regulatory element binding protein-2 (SREBP-2) as well GAPDH (as a housekeeping gene)] were performed by using the mastercycler gradient (Eppendorf). Approximately 30–40 cycles of amplification were used at 95°C for 30 s, 58°C for 30 s, and 72°C for 30 s. Amplicons were visualized on standard ethidium bromide-stained agarose gels. Importantly, we have established the experimental conditions relative to RT-PCR, which correspond to the linear portion of the exponential phase for every gene expression.

### Statistical Analysis

All values were expressed as the mean ± SD. The data were evaluated by ANOVA where appropriate, and the differences between the means were assessed using the Dunnett’s post test. A *P* value <0.05 was considered statistically significant.

## Results

### PYY and Cell Integrity

Before starting the evaluation of PYY effects on lipid homeostasis, it was mandatory to determine that this gastrointestinal peptide does not disturb cell viability and monolayer formation. As assessed by trypan blue exclusion, cell viability was not affected (data not shown). Moreover, measurement of transepithelial resistance, alkaline phosphatase, and sucrase activity did not disclose any significant perturbation in mucosal barrier function and cell differentiation (data not shown). Therefore, it could be concluded that PYY does not exert any cytotoxic effects on Caco-2/15 cells.

Since various investigators have reported the regulation of PYY output by lipids, it was important to assess that the cellular model Caco-2/15 also responds to these stimuli. Indeed, PYY was positively stimulated by fatty acids as shown in Figure 1. However, the addition of fatty acids to the basolateral medium resulted in a higher PYY output than fatty acids administered to the apical compartment.

RETRACTED

**Figure 1:** Influence of oleic acid on PYY secretion in the apical and basolateral media. Oleic acid at the concentrations of 0.7 mM and 1.4 mM was added either to the apical or basolateral medium. Following the 2-h incubation period, both apical and basolateral media were assessed for their PYY content. Values are expressed as means ± SD for n = 3 separate experiments in each group. CTR, Control; Baso, basolateral; OA, Oleic Acid.

### Localization of PYY Receptor in Caco-2/15 Cell Line

When seeded on porous filters (Transwell), Caco-2/15 cells allow access to both sides of the bipolar intestinal epithelium. Therefore, it is possible to explore the role of PYY in the regulation of lipoprotein secretion as a function of PYY site delivery: apical and basolateral compartments corresponding to intestinal lumen or serosal circulation, respectively. However, it was important to first show whether NPY1R receptor is localized in the apical and the basolateral membrane. Therefore, both membranes were isolated as described in our previous studies [36]–[38]. Careful scrutiny was carried out to assess the purity of the brush-border and basolateral membranes and to exclude the contamination by other organelle membranes. First, brush-border membrane (BBM) purity was determined by assessing the enrichment of specific brush-border markers, such as sucrase/isomaltase. Western blot analysis showed that the protein mass of this enzyme was increased by a factor of 55–62.5 in isolated intestinal BBM in comparison with homogenates of intestinal mucosa or Caco-2/15 cells (data not shown). Second, the typical microvillus carcino-embryonic antigen was enriched 7.0- to 8.2-fold in BBM (data not shown). Third, we excluded contamination by the endoplasmic reticulum and the Golgi by measuring the activity of glucose 6- phosphatase and galactosyltransferase, respectively, which were undetectable in BBM. Forth, Na+/K+-ATPase, a classical basolateral protein, was detectable only in basolateral membranes and not found in BBM (data not shown).

Following purification and purity assessment, Western blot analysis, using a specific antibody, indicates the presence of Y1 receptor in both the apical and basolateral membranes (Figure 2). However, the receptor protein mass was preponderant in the basolateral membrane. Given the distribution of the receptor on both sides of the Caco-2/15 cells, we decided to investigate its actions by adding PYY separately to apical and basolateral compartments.

**Figure 2:** Detection of Y1 receptor (NPY1R) in Caco-2/15 cells in culture. Following differentiation, Caco-2/15 cells were homogenized and apical and basolateral membranes were isolated. Aliquots were fractionated by SDS-PAGE and electrotransferred onto nitrocellulose membranes. The blots were then incubated with the polyclonal antibody overnight at 4°C. Immunocomplexes were revealed by means of horseradish peroxidase-conjugated goat anti-rabbit immunoglobulin and an enhanced chemiluminescence kit. Y1 receptor mass was quantitated by use of an HP Scanjet scanner equipped with a transparency adapter and software. Values are expressed as means ± SD for n = 3 separate experiments in each group.

RETRACTED

### Effect of PYY on Apical Cholesterol Uptake

Following pre-incubation (24 h) of Caco-2/15 cells with medium containing 50 nM and 200 nM of PYY, we determined how the addition of PYY to either the apical or basolateral compartment modifies cholesterol uptake. As illustrated in Figure 3, only the addition of PYY to the apical compartment was able to lower the capacity of Caco-2/15 cells to incorporate cholesterol.

**Figure 3:** Effects of the administration of PYY (1–36) to the apical or basolateral medium on cholesterol uptake in Caco-2/15 cells. Differentiated Caco-2/15 cells were cultured for 24 h in MEM containing 50 nM or 200 nM of PYY in their apical or basolateral medium, in the presence of 100 µM cholesterol in apical (with 250 000 dpm [^14^C]-cholesterol). Data are reported as % of control values representing 100%. Values represent the mean ± SD for n = 3 separate experiments in each group. * P<0.05 vs. controls, ** P<0.01 vs. controls.

### Influence of PYY on Cholesterol Protein Transporters

The decrease in cholesterol uptake exhibited by Caco-2/15 cells exposed apically to PYY may be due to differences in the expression of cholesterol transporters. To test this hypothesis, the protein expression of cholesterol transporters (NPC1L1, SR-BI and CD36) was examined by Western blot. As shown in Figure 4, the apical addition of PYY at the two concentrations (50 and 200 nM) resulted in a significant decrease in the protein expression of NPC1L1 without any changes in SR-BI and CD36. Besides, no alterations in all these cholesterol transporters were noted when PYY was delivered to the basolateral medium. Since ABCG5 and ABCG8 restrain cholesterol absorption in the lumen of the intestine by excreting absorbed cholesterol, it was mandatory to assess their protein expression in response to PYY administration. Figure 5 shows no alterations in the protein mass of ABCG5 and ABCG8 following PYY inclusion either in the apical or basolateral compartments.

**Figure 4:** Effects of the administration of PYY (1–36) to the apical or basolateral medium on the protein expression of transporters mediating cholesterol absorption. Caco-2/15 cells were cultured for 24 h in MEM as described in the legend of Figure2. Western blot was used to analyze the protein expression of NPC1L1 (A), SR-BI (B) and CD36 (C). Values are means ± SD for n = 3 separate experiments in each group and are reported as % of control values representing 100%. *P<0.01 vs. controls.

RETRACTED

**Figure 5:** Effects of the administration of PYY (1–36) to the apical or basolateral medium on the protein expression of ABCG5 and ABCG8. Caco-2/15 cells were cultured for 24 h in MEM as described in the legend of Figure 2. Western blot was used to analyse the protein expression of ABCG5 (A) and ABCG8 (B). Data represent means ± SD for n = 3 separate experiments in each group and are reported as % of control values representing 100%.

### Effects of PYY on *De novo* Cholesterol Synthesis

Experiments were performed to examine the regulatory role of PYY on newly intracellular cholesterol synthesis. Caco-2/15 cells were, therefore, incubated with [^14^C]-acetate for 24 h and the two free and esterified forms of cholesterol were analyzed by TLC. Apical and basolateral administration of PYY at the largest concentration slightly enhanced the synthesis of free and esterified cholesterol (Figure 6). Interestingly, the delivery of PYY to the basolateral compartment was more effective in raising cholesterol formation.

**Figure 6:** Effects of the administration of PYY (1–36) to the apical or basolateral medium on cholesterol synthesis. After 24 h incubation with [^14^C]-acetate, cells were homogenized. Lipids were extracted in chloroform/methanol and separated by TLC. The free cholesterol (FC) and cholesteryl ester (CE) bands were scraped off the plate and counted. Data represent means ± SD for n = 3 separate experiments in each group. *P<0.05 vs. controls, **P<0.01 vs. controls.

### PYY and the Key Regulatory Proteins of Cholesterol Metabolism

Next, we determined the impact of PYY on the regulatory sterol enzymes: HMG-CoA-R, the rate-limiting step in cholesterol synthesis, and ACAT-2, an integral protein present in the rough endoplasmic reticulum that catalyzes the formation of cholesteryl ester from free cholesterol. HMG-CoA-R protein expression increases with only the addition of 200 nM PYY to the basolateral medium (Figure 7A). Moreover, the same concentration of PYY at the same delivery site displayed a trend of decrease in HMG-CoA-R phosphorylation, which reflects an activation of the enzyme (Figure 7B). Confirmatory data were obtained when the P-HMG-CoA reductase/HMG-CoA reductase ratio was calculated (Figure 7C). As to ACAT-2, while the apical addition of PYY remained without effect on its protein mass, a significant decrease was noted with in the protein expression with the highest PYY concentration administered in the basolateral compartment (Figure 8). Finally, we tested the effects of LDLR and could not find a significant impact of PYY administration to the apical and basolateral media (Figure 9).

RETRACTED

**Figure 7:** Effects of the administration of PYY (1–36) to the apical or basolateral medium on the protein expression of HMG-CoA-R (A) and phosphorylated HMG-CoA-R (B). Caco-2/15 cells were cultured for 24 h in MEM as described in Figure 2. Western blot was used to analyze the protein expression and phosphorylation of HMG-CoA-R. Values are means ± SD for n = 3 separate experiments in each group and are reported as % of control values representing 100%. *P<0.05 vs. controls, ** P<0.01 vs. controls.

**Figure 8:** Effects of the administration of PYY (1–36) to the apical or basolateral medium on the protein expression of ACAT-2. Caco-2/15 cell line was cultured for 24 h in MEM described in Figure 2. Western blot was used to analyze the protein expression of ACAT-2. Values are means ± SD for n = 3 separate experiments in each group and are reported as percent. *P<0.01 vs. controls.

**Figure 9:** Effects of the administration of PYY (1–36) to the apical or basolateral medium on the protein expression of LDL-receptor (LDL-R). Caco-2/15 cells were cultured for 24 h in MEM as described in the legend of Figure 2. Western blot was used to analyse the protein expression of LDL-R. Data represented means ± SD for n = 3 separate experiments in each group and are reported as % of control values representing 100%.

### PYY and Lipoprotein Production

The ability of Caco-2/15 cells to assemble and secrete lipoproteins was assessed as a function of PYY concentrations. Figure 10 shows little effect of PYY on the production of lipoproteins. Nevertheless, a small decrease in CM output was noted with the addition of 200 nM to the basolateral medium (Figure 10A). The same trend was observed in LDL with the administration of 200 nM to the apical medium (Figure 10C). However, no alterations were noted in VLDL (Figure 10B) and HDL (Figure 10D).

**Figure 10:** Effects of the administration of PYY (1–36) to the apical or basolateral medium on lipoproteins output. Differentiated Caco-2/15 cells were cultured for 24 h in MEM containing 50 nM or 200 nM of PYY in their apical or basolateral medium, in the presence of [^14^C]-oleic acid for 24 h. Thereafter, the media were ultracentrifuged to isolate lipoproteins at their specific densities. Radioactivity incorporated into each fractions was further determined. Data were analyzed as dpm/mg of total protein but were reported as percent difference relative to control. Data represent means ± SD for n = 3 separate experiments in each group. * P<0.05 vs. controls. CM**;** Chylomicrons (A), VLDL; Very-low density lipoprotein (B), LDL; low density lipoprotein (C) and HDL; high density lipoprotein (D).

RETRACTED

### PYY and Apolipoprotein Biosynthesis

In attempt to explore whether PYY influences the synthesis and secretion of apos, the gastrointestinal peptide was added either to the apical or basolateral compartment in combination of [^35^S]-methionine as a precursor of peptide elongation. Only the biogenesis of apo A-I was increased with the apical addition of 50 nM PYY. On the other hand, the addition of PYY to the basolateral compartment was more effective in reducing the synthesis of apos B-48 and B-100 (Figure 11).

**Figure 11:** Effects of the administration of PYY (1–36) to the apical or basolateral medium on the synthesis of apolipoproteins (apo). Epithelial cells at 14 days post-confluence were incubated with [^35^S]-methionine in the presence of PYY (1–36) (50 or 200 nM) and unlabeled oleic acid for 24 h to stimulate apo biogenesis. At the end of the labelling period, cells were washed, homogenized, and centrifuged. Supernatants from the cell homogenates were then reacted with excess antibodies for 18 h at 4°C to precipitate specific apos. Immune complexes were washed and analyzed by linear 4–15% SDS-PAGE. After electrophoresis, gels were sliced and counted for radioactivity. Data represent means ± SD for n = 3 separate experiments in each group. Values are reported as % of control values representing 100%. *P<0.05 vs. controls.

### PYY and Microsomal Trigyceride Transfer Protein

MTP has been identified as a crucial protein for intracellular apo B lipoprotein assembly. We have, therefore, determined the influence of PYY on its protein expression. No significant changes were noticed in the protein mass assessed by Western blot between controls and cells treated with PYY(1–36). However, there was a divergence between apical and basolateral compartments (Figure 12).

**Figure 12:** Effects of the administration of PYY (1–36) to the apical or basolateral medium on the protein expression of MTP. Caco-2/15 cells were cultured for 24 h in MEM as described in the legend of Figure 2. Western blot was used to analyse the protein expression of MTP. Data represent means ± SD for n = 3 separate experiments in each group and are reported as % of control values representing 100%. * P<0.05 vs. 50 nM or 200 nM in apical side.

### PYY and Transcription Factors

To approach the mechanisms triggered by PYY, we assessed the gene expression of several factors that affect the transcription of a variety of genes associated with lipid and cholesterol metabolism, including RXR(α, β), liver LXR(α, β), PPAR(α, β, γ), and SREBP-2. Data on Figures 13 and 14 illustrate how PYY at the concentrations of 50 and 200 nM impacted on the expression of the different nuclear and transcription factors in Caco-2/15 cells. It did not cause any significant variation on the mRNA levels of RXRβ (Figure 13B), LXRα (Figure 13C), LXRβ (Figure 13D), and PPARγ (Figure 14C), whereas it produced a significant reduction in gene expression of RXRα (Figure 13A), PPARα (Figure 14A) and PPARβ (Figure 14B) in Caco-2/15 cells incubated with 200 nM PYY in basolateral medium. Finally, when we explored the effect of PYY on SREBP-2 gene expression, we detected a significant enhancement upon exposure to 50 nM or 200 nM PYY in apical compartment (Figure 14D).

RETRACTED

**Figure 13:** Effects of the administration of PYY (1–36) to the apical or basolateral medium on RXR and LXR gene expression in Caco-2/15 cells. PCR analysis was performed on Caco-2/15 cell line at 14 days post-confluence to analyze mRNA of RXRα (A), RXRβ (B), LXRα (C), LXRβ (D). Values represent means ± SD for n = 3 separate experiments in each group and are reported as % of control values representing 100%. *P<0.05 vs. controls, **P<0.01 vs. controls.

**Figure 14:** Effects of the administration of PYY (1–36) to the apical or basolateral medium on PPAR and SREBP-2 gene expression in Caco-2/15 cells. PCR analysis was performed on Caco-2/15 cell line at 14 days post-confluence to analyze mRNA of PPARα (A), PPARβ (B), PPARγ (C), SREBP-2 (D). Values represent means ± SD for n = 3 separate experiments in each group and are reported as percent difference relative to control. * P<0.05 vs. controls, **P<0.01 vs. controls.

## Discussion

PYY exerts anorexigenic effects via satiety signalling actions in the brain and the periphery. It is known that PYY regulates intestinal motility [39], [40] and prolonged gastric emptying [41]. Surprisingly, little information is available, to our knowledge, on the role of PYY in intestinal cholesterol uptake, synthesis and transport by lipoproteins in the small intestine. For the first time, our work has attempted to unravel the role of PYY in cellular cholesterol metabolism. Our data indicate that PYY could decrease cholesterol uptake by reducing the protein mass of NPC1L1, an essential protein for dietary cholesterol absorption. PYY also elicited cholesterogenesis by translational regulation of HMG-CoA-R. Small negative effects of PYY were noted on CM and LDL along with alterations of certain types of apo. Finally, PYY was able to regulate specific transcription factors implicated in the regulation of lipid and cholesterol metabolism. Importantly, the effects of PYY were noted to depend on two factors in intestinal cells: the PYY site of administration (apical vs. basolateral) and PYY concentrations (50 vs. 200 nM).

RETRACTED

**Figure 15:** Integrative scheme documenting the asymmetrical regulation of lipid transport by apical and basolateral PYY stimuli using differentiated, polarized Caco-2/15 cells.

Influences of apical and basolateral domains of the enterocyte, which correspond to the intestinal lumen and the serosal circulation, respectively, are actually limited. Indeed, there are only few studies dealing with the stimuli, including PYY, originating from apical and basolateral compartments. Some investigators have also detected distinct effects on various targets depending on the stimulus location. For example, addition of transforming growth factor beta (TGF-β) to the basolateral medium resulted in phosphorylation of the intracellular protein signalling Smad2, whereas no phosphorylation was observed when TGF-β was added to the apical chamber [42]. According to the authors, there are elements of communication between epithelial and mesenchymal in polarized epithelia, which allow vectorial signalling. Furthermore, intestinal epithelial cells were capable of organizing their response to inflammatory signals and producing inflammatory mediators in a bidirectional, vectorial fashion [43]. Finally, we have recently shown that there is a discrete regulation of SR-BI from stimuli, originating from apical and basolateral media, such as n−3 and n−6 fatty acids, fibrate, cholesterol, 7-ketocholesterol, methyl β-cyclodextrin, lipopolysaccharide, tumor necrosis factor-α, interferon γ, insulin, growth hormone and epidermal growth factor [44]. It is the first time that vectorial response in link with PYY location has been treated. Interestingly, we have added new studies evaluating how FAs regulate the secretion of PYY from the apical and basolateral media (Figure 1). Our experiments showed that oleic acid at the concentration of (1.4 mM), administred to the basolateral medium, upregulated PYY output from the basolateral pole. This increased output was higher than that caused by the stimulation of apical PYY secretion, by oleic acid at the same concentration. Interestingly, these observations are in line with data from Figure 2 illustrating the preponderance of receptor protein mass in the basolateral membrane.

To evaluate the involvement of PYY in cholesterol homeostasis, we used the Caco-2/15 cell line that undergoes a process of spontaneous differentiation leading to the formation of a monolayer of cells expressing several morphological and functional characteristics of the mature enterocyte. This remarkable intestinal model is regarded as the most appropriate for the investigation of gut absorption and interactions, nutrition, toxicology food microbiology, bioavailability tests, and screening of drug permeability in discovery programs. Multiple studies from our laboratory [21], [29], [30], [32]–[35], [38] and from other groups have shown that Caco-2/15 monolayers are fully appropriate for the study of lipid/lipoprotein homeostasis. Importantly, when seeded on porous filters (Transwell), Caco-2/15 cells allow access to both sides of the bipolar intestinal epithelium. Therefore, we were able in the present work to explore the regulation of cholesterol metabolism as a function of PYY site delivery: apical and basolateral compartments corresponding to intestinal lumen or serosal circulation, respectively. As a prerequisite to our study, it was necessary for us to demonstrate the presence of PYY receptor in Caco-2/15 cells and its distribution on both sites (apical and basolateral membrane), thus favouring binding of the ligand (PYY) and its internalization [45]. Importantly, L cells in the intestinal epithelium secrete PYY (1–36) into the lumen of the intestine across the apical membrane and the blood circulation via the basolateral membrane [22]–[24]. The presence of PYY in the apical and basolateral membranes may be dependent on the type of nutrient ingested and may serve to modulate the diverse physiologic roles of PYY. Moreover, the concentrations of PYY are variable in the circulation depending on the physiological states: they are low during fasting and significantly increase after meal consumption, reaching a plateau following 2 h post-prandially.

RETRACTED

In the current research, we used human PYY(1–36) instead of PYY(3–36), since previous reports have shown the stimulation of apo A-IV by PYY(1–36) in Caco-2/15 cells [46]. According to the authors of this paper, only Y1 receptor mediated this stimulatory effect following binding with the PYY (1–36) ligand given that the other Y2 and Y5 receptors for PYY (3–36) seemed not operational in view of their undetectable mRNAs in Caco-2/15 cells. In these studies, the concentrations of PYY reached 200 nM in order to obtain the stimulation of Apo A-IV. Additionally, the PYY (1–36) was repeatedly used in studies associated with lipid metabolism in the intestine [12], [15], [47]. Finally, in terms of cell differentiation, maintenance of the intestinal epithelium and the regulation of absorption in the intestine, investigators have largely turned to the PYY (1–36), which has a high affinity for the receptor NPY1R [48]. Accordingly, the presence of the receptor NPY1R has already been noted in previous studies using intestinal Caco-2/15 cells. Taking into account the secretion of PYY from both apical and basolateral compartments of the enterocytes [22], [49], it appeared important for us to determine the status of this receptor both in apical and basolateral sides.

In the present work, PYY was used in the 50–200 nM range, since numerous investigators reported plasma concentrations of PYY in the range of pM to nM [50]. But these concentrations could considerably be augmented following exercise and meal tests [51], [52]. Additionally, levels of PYY varied according to the intestinal region and reached values of ∼1000 pmol/g colonic or rectal tissue [53], [54]. Therefore, given these collective data, we do not think that PYY was employed in high pharmacological doses in our studies.

NPC1L1 has been identified at the surface of plasma membrane as a critical protein in the exogenous cholesterol absorption [55]. It transports cholesterol from the lumen into enterocytes where intestinal ACAT-2 then converts cholesterol to CE that is packed into CM. SR-BI and CD36 are also located on the brush border membrane and can contribute to the absorption of cholesterol. Our experiments showed an inhibition of cholesterol uptake with the addition of PYY to the apical medium, which was confirmed by NPC1L1 downregulation, but SR-BI and CD36 remained unaffected. To approach the underlying mechanisms, we analyzed the gene expression of specific transcription factors involved in cholesterol homeostasis. We first examined PPARs that represent a subgroup of the nuclear receptor superfamily, including PPAR(α, β, γ) heterodimerizing with the RXR and, upon ligand binding, become transcriptionally active and control a series of genes of lipid and energy metabolism. Even if previous studies showed that specific activation of PPARα and PPARβ decreases cholesterol absorption via an inhibitory effect on NPC1L1 expression in the proximal small intestine [56], , no significant differences were noted, in our study, in the gene expression of apical PPARα and PPARγ in contrast with a substantial decrease in PPARβ mRNA. These findings are not consistent with an implication of PPARs in PYY-mediated NPC1L1 downregulation. We then turned to LXRs that act as oxysterol sensors of intracellular cholesterol homeostasis [58]. LXRs form obligate heterodimers with RXRs, which activate their target genes by binding to specific response elements (LXREs). Recently, it has been revealed that LXRs seem to govern dietary cholesterol fate in the enterocyte by downregulating apical absorption through NPC1L1 [59]. Our data displaying no changes in LXRα,β and decreased RXRα are not lining up with a possible involvement of these transcription factors in PYY-mediated NPC1L1 downregulation. Finally, the upregulation of SREBP-2 gene expression in response of PYY could not explain the reduction in cholesterol transport and in NPC1L1 protein abundance. An important direction to follow in next studies in order to detect the mechanisms of action of PYY will consist in investigating the formation of NPC1L1–flotillins-positive cholesterol-enriched membrane microdomains. In fact, NPC1L1 performs the task of apical cholesterol uptake by collaborating with flotillins to form cholesterol-enriched membrane microdomains. Internalization of these membrane microdomains brings a large amount of cholesterol into the cells which might be a mechanism accounting for high efficiency of cholesterol absorption [60].

RETRACTED

In our studies, HMG-CoA R expression was found to be 3-fold upregulated, but the cholesterol synthesized was only increased 1.2 fold in response to the PPY. In fact, HMG-CoAR can be regulated through alterations of its quantity and/or of its catalytic efficiency. In particular, mechanisms implicated in the regulation of HMG-CoAR include the manipulation of enzyme quantity through transcriptional [61], [62] and post-transcriptional processes [63], [64] and enzyme degradation [65], [66], as well as the alteration of enzyme catalytic activity by membrane composition and fluidity [67], by thiols [68], by microtubules [69], or by cytosolic lipid inhibitors and their binding proteins [70]. It is, therefore, possible that despite the increase in HMG-CoA-R mass, PYY may elicit another regulatory mechanism, e.g. the reversible inactivation and reactivation of HMG-CoA-R via its covalent phosphorylation and dephosphorylation.

Interestingly, the addition of PYY to the basolateral medium resulted in a significant decrease in the biogenesis of apo B-48, an essential protein in the assembly of TG-rich lipoprotein. A slight, but significant, decrease was also observed in CM output. It is generally accepted that the intracellular mechanism of TG-rich lipoprotein assembly requires apo B synthesis and association. An early step in this process is the cotranslational lipidation of apo B that is transiently bound to the endoplasmic reticulum membrane where it is folded. The addition of lipids stabilizes apo B-48 and prevents its proteolytic degradation via the ubiquitin-dependent proteasomal pathway [71], [72]. It is therefore reasonable to suggest that the defective synthesis of CM in Caco-2/15 cells, supplemented in their basolateral medium with PYY, is due to limited apo B-48 protection from misfolding and degradation despite MTP protein expression enhancement, which does not reflect MTP activity or alternatively could not compensate for the marked apo B-48 proteolytic degradation by the proteasome. Finally, although the decrease of CM appears modest despite the statistical significance, it is reasonable to propose that PYY can affect the intestinal transport of lipids given the significant length of the intestine and especially the perpetual postprandial state characterizing nowadays the Western population, which is actually subjected to abundant and frequent feeding.

RETRACTED

This study shows interesting results in relation with the influence of PYY on intestinal cholesterol metabolism. Previous reports documented that binding of PYY to its receptors resulted in inhibition of electrolyte secretion [49], [73] via inhibition of cAMP production [74] suggesting that PYY was likely to exert its effect through an inhibition of adenylyl cyclase. At this time, we have no evidence as to the role of cAMP in PYY-mediated regulation of cholesterol metabolism. However, the present data point out that PYY in the apical compartment can essentially decrease cholesterol uptake through the downregulation of NPC1L1, while basolateral PYY can reduce the output of CMs via a decrease in apo B-48 biosynthesis. More *in vivo* and *in vitro* studies are absolutely required to determine the specific endocrine and paracrine mechanisms triggered by PYY for the regulation of the transport of various nutrients.

Although the PYY receptor is more concentrated on the basolateral membrane vs. the apical membrane, only the administration of PYY apically was able to decrease cholesterol uptake. This intriguing finding may be explained by distinct intracellular signalling pathways or discrete regional regulation at the two intestinal poles, triggered by the two PYY receptors located on basolateral and apical membranes. In previous studies, fasting PYY correlated negatively with plasma total cholesterol, LDL-cholesterol and HDL-cholesterol in response to bariatric surgery in severely obese patients [19] and overfeeding in normal weight subjects [20]. Our data indicate for the first time that PYY may act on the intestine to down-regulate cholesterol absorption, which may influence cardiovascular risk factors.

Although most early studies so far have been concerned by the concept that factors secreted from the gut endocrine system participate in the regulation of gastrointestinal functions, growing evidence underlines their functions in metabolic pathways and in the pathophysiology of various metabolic diseases, including obesity, insulin resistance and diabetes, which lead to cardiovascular diseases. Indeed, a great number of gastrointestinal peptides, including PYY affect numerous organs while modulating energy storage, lipolysis, body weight, appetite, satiety, β-cell preservation and glucose metabolism [75]. Recently, it has been shown that the gut plays a major role in glucose homeostasis via the regulation of both insulin secretion and sensitivity [76]–[78], while bariatric surgery likely influences several GI pathways in complementary ways to improve glucose control and diabetes. Accordingly, the selective activation of the neuropeptide Y receptor by PYY (3–36) suppresses appetite, reduces acute food intake, causes body weight loss and provides a promising approach to obesity management. Therefore, the control of receptor Y by PYY becomes an attractive mechanism for the therapeutic management of obesity and its associated morbidities such as insulin resistance and diabetic dyslipidemia. Limited studies are available on the effects of PYY on cholesterol metabolism, but indirect evidence points to this important issue. As an example, two obese women groups differed from lean controls by showing lower plasma PYY (3–36) both under basal conditions and after meal, and this was accompanied by higher postprandial blood glucose and insulin levels, as well as total cholesterol and LDL-cholesterol [79]. Furthermore, with the sustained rise in GLP-1 and PYY levels, there was a decline in glucose, insulin, total cholesterol, LDL-cholesterol, and triglyceride levels [80]. In another investigation, long-term exercise training displayed beneficial effects for overweight adolescents with respect to the increase in PYY, decrease in TG and lowering of total cholesterol and LDL-cholesterol although the changes of the cholesterol variables did not reach statistical significance [81]. In another study, overfeeding significantly raised fasting PYY, which was negatively correlated with the changes of total cholesterol, HDL and LDL while being positively associated with HDL cholesterol [20]. Altogether, the information obtained from these research groups indicates an indirect link between PYY and lipid (cholesterol and triglyceride) metabolism. As to the relationship between PYY and cardiovascular diseases, various investigators reported that the beneficial effects of dietary feeding (e.g. diminution of postprandial glycemia, lipidemia and insulinemia along with the reduction of cardiovascular disease risks) could be due to its actions on the levels of PYY among many peptides [82]. In addition, Hanusch-Enserer et al. concluded that, in restrictive bariatric surgery, PYY correlates with major cardiovascular risk factor and surrogate parameters of insulin secretion [19]. Finally, according to Zwirska-Korczala et al., down-regulation of PYY secretion may lead to progression of endothelial dysfunction and may promote acceleration of atherosclerosis [51]. Nevertheless, additional studies are needed to scrutinize this important aspect and to evaluate cause-effect evidence of PYY and cardiovascular risk factors.

RETRACTED

However, it is important to note that, following binding with PYY, Y1 receptors rapidly internalize through clathrin-coated pits and recycle back to the plasma membrane [83], [84]. It remains unknown whether these internalized receptors enter a recycling pathway leading to relocalization at the cell surface.

In summary, our data suggest that PYY may exert an impact on intracellular lipid metabolism depending on the route of administration as well illustrated in Figure 15. Although it is known that, following binding with PYY, Y1 receptors rapidly internalize through clathrin-coated pits and recycle back to the plasma membrane, no information is available to indicate whether internalized PYY may be transferred from one membrane to another, which may influence the effects of PYY on one specific pole of the cell. Further investigations are required to explore this exciting issue. For now, our efforts at least highlighted a segregation in the function of PYY in the two cell poles: (i) at the apical compartment, it decreased LDL secretion and lowered cholesterol uptake via the down-regulation of NPC1L1 transporter, while it enhanced certain types of apos and cholesterogenesis; and (ii) at the basolateral compartment, it disclosed ability to augment cholesterol synthesis and to lower chylomicron output through the lowering of apos and transcriptional factors. More work is necessary to further establish the role and mechanisms action of PYY in lipid transport in the enterocytes.
